# Long non-coding RNA ANRIL promotes the invasion and metastasis of thyroid cancer cells through TGF-β/Smad signaling pathway

This article has been retracted.

**DOI:** 10.18632/oncotarget.11087

**Published:** 2016-08-05

**Authors:** Jian-Jie Zhao, Shuai Hao, Ling-Li Wang, Chun-Yan Hu, Shu Zhang, Ling-Ji Guo, Gang Zhang, Bo Gao, Yan Jiang, Wu-Guo Tian, Dong-Lin Luo

**Affiliations:** ^1^ Department of Breast, Thyroid, and Vascular Surgery, Research Institute of Surgery, Daping Hospital, Third Military Medical University, Chongqing, 400042, P. R. China

**Keywords:** long non-coding RNA ANRIL, thyroid cancer, p15I^NK4b^, TGF-β/Smad signaling pathway, TPC-1

## Abstract

**Objective:**

To investigate the effect of antisense non-coding RNA in the INK4 locus (ANRIL) on invasion and metastasis of thyroid cancer (TC).

**Results:**

ANRIL expression was significantly up-regulated in TC tissues and cells (*P <* 0.001), and ANRIL expression was significantly different regarding histological grade and LNM (both *P <* 0.01). The siRNA-mediated ANRIL silencing inhibits proliferation, invasion, and metastasis of TPC-1 and SW579 cells, and lung metastasis, which can be reversed by TGF-β1 siRNA. The mRNA levels of p15^INK4b^, p14^ARF^ and p16^INK4a^ in TPC-1 and SW579 cells increased significantly after silencing ANRIL (all *P <* 0.001), and TGF-β1 siRNA could reverse the ANRIL siRNA induced increase of p15INK4b; expressions of TGF-β1 and p-Smad2/3 were increased after silencing ANRIL (both *P <* 0.05).

**Materials and methods:**

TC and adjacent normal tissues were collected from 105 TC patients. LncRNA ANRIL expressions were detected by qRT-PCR. The siRNA ANRIL and siRNA TGF-β1 were constructed for TPC-1 and SW579 cell line transfection: si-ANRIL group, si-TGF-β1 group, si-ANRIL + si-TGF-β1 group, negative control group and blank group. Effects of ANRIL silencing on proliferation, invasion and metastasis of TC cells was detected by MTT assay, Transwell assay and tail vein injection of nude mice *in vitro* and *in vivo*. TGF-β1 and p-Smad2/3 expressions in TGF-β/Smad signaling pathway were detected by western blot.

**Conclusions:**

ANRIL may reduce p15^INK4B^ expression through inhibiting TGF-β/Smad signaling pathway, promoting invasion and metastasis of TC cells, and the silencing of ANRIL inhibits the invasion and metastasis of TPC-1 cells.

## INTRODUCTION

Thyroid cancer (TC) is originated from follicular or parafollicular thyroid cells. Globally, TC shows an increasing trend and results in 36,000 deaths in 2010 compared to 24,000 in 1990; however, with effective treatment, the five-year survival rate of TC is still low [1, 2]. TC incidence has been increased by an average of 4.5% per year from 2007 to 2011 in United States, and TC ranks the eighth most frequent cancer in China, thus the rapid increase in TC incidence poses a substantial burden [3–5]. TC is considered as a multicausal disease related to multiple environmental and genetic predisposing factors, such as environmental exposure to ionizing radiation, obesity, and genetic and epigenetic alterations, but significant uncertainty remains regarding its causes [6, 7]. Long non-coding RNAs (lncRNA) are non-protein coding transcripts with more than 200 nucleotides, and up- or down-regulated lncRNA expressions in cancers suggests a major contributor role of aberrant lncRNA expression in carcinogenesis [8]. Further, it has been previously reported that a highly thyroid-specific lncRNA might play potential roles in the occurrence and development of TC with dramatically altered expression [9].

LncRNAs, acting as markers of cell fate and parental imprinting, are involved in a number of regulatory functions such as modulating apoptosis and invasion, and reprogramming induced pluripotent stem cells [10, 11]. LncRNAs play crucial roles in epigenetic gene regulation, transcriptional control and post-transcriptional regulation, and RNA based epigenetic regulatory network, through small interfering RNAs (si-RNA), has implications in both cellular and pharmacology evolution [12, 13]. Antisense non-coding RNA in the INK4 locus (ANRIL), also known as CDKN2B-AS, is a lncRNA consisting of 19 exons, spanning 126.3kb in the genome. ANRIL is located within the p15/CDKN2B-p16/CDKN2A-p14/ARF gene cluster at chromosome 9p21 in the antisense direction [14]. It has been previously documented that ANRIL binds to chromobox 7 (CBX7) and to SUZ12, and is involved in transcriptional repression through these interactions. In addition, and associations between altered expression of ANRIL and various cancers have been reported to help understand molecular pathogenesis [15–17]. ANRIL is thought to be a possible oncogene in bladder cancer and positively regulates bladder cancer cell proliferation and apoptosis through the intrinsic apoptosis pathway [18]. In addition, significant roles of ANRIL have been found in the development of esophageal squamous cell carcinoma (ESCC) by inhibiting p15 (INK4b) through the transforming growth factor β1 (TGF-β1) signaling pathway [19]. Importantly, great progress has been achieved in understanding the molecular pathogenesis of TC, as best exemplified by the elucidation of the fundamental role of several major signaling pathways and related molecular derangements [20]. TGF-β restrains the proliferation of many human cell lines and tissues including thyroid, and a major role of TGF-β/Smad signaling has been suggested in the induction of epithelial-mesenchymal transition (EMT) in TC cells [21, 22]. We hypothesized that ANRIL might also play a role in the development of TC through the TGF-β/Smad signaling pathway. However, few studies were performed on the both roles of ANRIL and TGF-β/Smad signaling pathway in TC. Therefore, in the present study, the expression of ANRIL in TC tissues/cell lines and adjacent normal tissues/normal thyroid cell line are detected; additionally, the effect and mechanism of ANRIL on the invasion and metastasis of TC was evaluated by silencing ANRIL with si-RNA and involvement in the TGF-β/Smad signaling, to clarify the role of ANRIL and TGF-β/Smad signaling pathway and the association between ANRIL and TGF-β/Smad signaling pathway in TC.

## RESULTS

### Expression of ANRIL and its relationship with clinicopathological features

The results of qRT-PCR showed significantly higher expression of ANRIL mRNA in the TC tissues relative to the adjacent normal tissues (*P* < 0.001) (Figure 1). The 105 TC patients were divided into high expression group (≥ mean relative expression of ANRIL) and low expression group (< mean relative expression of ANRIL) based on the mean relative expression of ANRIL in the TC tissues. ANRIL mRNA expression showed no significant difference regarding gender, age, pathological type, tumor volume, multicenteric cancer foci or surgical procedure (all *P* > 0.05), but there was a significant difference in ANRIL mRNA expression for tumor node metastasis (TNM) staging and LNM (both *P* < 0.01) (Table 1).

**Figure 1:** The expression of ANRIL in thyroid cancer tissues and adjacent normal tissues detected by qRT-PCR; **P < 0.0001 qRT-PCR, quantitative real-time polymerase chain reaction

**Table 1:** Correlation between ANRIL and TGF-β1 expression and clinicopathological characteristics in thyroid cancer

Clinic parameter	ANRIL		Chi-square test *P* value	TGF-β1		Positive rate (%)	Chi-square test *P* value
	High no.case	Low no.case		−	+		
Gender							
Male	18	20	0.632	10	28	73.68	0.700
Female	35	32		20	47	70.15	
Age							
≥ 45	37	30	0.196	21	46	68.66	0.404
< 45	16	22		9	29	76.32	
Pathological type							
Papillary adenocarcinoma	38	34	0.486	24	48	66.67	0.111
Follicular adenocarcinoma	15	18		6	27	81.82	
Tumor volume (cm)							
2~4	35	28	0.202	17	46	73.02	0.659
< 2	18	24		13	29	69.05	
Multicentric cancer foci							
Single	30	26	0.498	19	37	66.07	0.194
Multi	23	26		11	38	77.55	
Lymph node metastasis							
Yes	39	19	0.005	7	51	87.93	0.007
No	14	33		23	24	64.86	
Surgical procedure							
Subtotal thyroidectomy	33	31	0.781	22	42	65.63	0.100
Thyroidectomy	20	21		8	33	80.49	
Clinical stages							
I–II	13	32	< 0.001	18	27	80.00	0.025
III–IV	40	20		12	48	60.00	

### Expression of TGF-β1 in TC tissues

Immunohistochemically, TGF-β1 protein was mainly expressed in the cytoplasm, and presented with a diffused or granular yellowish-brown (Figure 2). Significantly lower positive rate of TGF-β1 protein expression was found in the adjacent normal tissues in comparison to the TC tissues [28.57% (30/105) vs. 71.43% (75/105), *P* < 0.001]. As showed in Table 1, the positive rate of TGF-β1 protein expression in TC patients without LNM was also lower compared with patients with LNM (64.86% vs. 87.93%, *P* = 0.010); patients with TNM staging I/II had significantly lower positive rate of TGF-β1 protein expression than patients with TNM staging III/IV (60.00% vs. 80.00%, *P* = 0.034). However, the positive rate of TGF-β1 protein expression was not related to age, gender, pathological type, tumor volume, multicenteric cancer foci or surgical procedure (all *P* > 0.05). Spearman correlation analysis showed that the ANRIL expression was positively correlated with the expression of TGF-β1 protein expression (*r* = 0.253, *P* = 0.004).

**Figure 2:** Expression of TGF-β1 protein in thyroid cancer (TC) tissues and adjacent normal tissues (× 200): TGF-β1 protein was mainly expressed in the cytoplasm, and presented with a diffused or granular yellowish-brown The positive rate of TGF-β1 protein expression in adjacent normal tissues was significantly lower than that in TC tissues.

### Expression of lncRNA ANRIL in cell line

qRT-PCR was used to detect lncRNA ANRIL expressions in K1, TPC-1 and SW579 and a strain of normal thyroid cells, Nthy-ori 3–1. The relative expressions of lncRNA ANRIL in K1 (4.07 ± 0.17), TPC (9.69 ± 0.28) and SW579 (5.90 ± 0.18) were higher than those in Nthy-ori 3–1 (3.02 ± 0.14) (all *P* < 0.0001). Since the expression of ANRIL was higher in TPC-1 and SW579 cell lines, TPC-1 and SW579 cell lines were used as model cells to study the function of ANRIL (Figure 3).

**Figure 3:** The expression of ANRIL in each thyroid cancer and normal thyroid cell lines detected by qRT-PCR; **, compared with Nthy-ori 3–1, P < 0.0001 qRT-PCR, quantitative real-time polymerase chain reaction.

### Effect of silencing ANRIL expression on the growth of TPC-1

The results of MTT and cell counting (Figure 4A–4B) showed that, compared with the blank group and the NC group, the cell growth was significantly inhibited in the si-ANRIL group (both *P* < 0.05); OD values showed no significant difference between the blank group and the NC group at each time point (all *P* > 0.05); OD value at time points of 24 h and 48 h were significantly higher in the si-TGF-β1 group and the si-ANRIL + si-TGF-β1 group than those of the blank group and the NC group (all *P* < 0.05). It was demonstrated that transfection of ANRIL siRNA significantly inhibited the growth of TPC-1 and SW579 cells, silencing TGF-β1 can promote the growth of TPC-1 and SW579 cells, and TGF-β1 siRNA can reverse the ANRIL siRNA induced inhibition of cell growth of TPC-1 and SW579.

**Figure 4:** The effect of lncRNA expression on the growth of thyroid cancer TPC-1 and SW579 cells detected by methyl thiazolyl tetrazolium (MTT) and cell counting (**A**) cell growth measured by MTT; (**B**) cell growth measured by cell counting; *, compared with blank group and NC group, *P* < 0.05.

### Silencing ANRIL expression inhibits TPC-1 and SW579 cell migration

The results of MTT showed that numbers of cells migrating through membranes of the blank group and were 74.8 ± 6.4 and 62.47 ± 5.26, the NC group were 72.5 ± 6.9 and 58.53 ± 5.74, respectively, without significant difference (*P* > 0.05). The numbers of cells migrating through membranes in the si-ANRIL group were 36.8 ± 5.8 and 22.17 ± 3.45, which was significantly lower than that of the blank group and the NC group (both *P* < 0.05). Therefore, silencing ANRIL can inhibit the migration of TPC-1 and SW579 cells. The numbers of cells migrating through membranes in the si-TGF-β1 group (112.4 ± 12.8 and 109.48 ± 9.52) was distinctively higher relative to the blank group and the NC group. The numbers of cells migrating through membranes in the si-ANRIL group (36.8 ± 5.8) were significantly lower than those in the si-ANRIL + si-TGF-β1 group (85.9 ± 11.8 and 76.58 ± 5.82) (all *P* < 0.05). The results indicated that exogenous low expression of TGF-β1 can promote TPC-1 and SW579 cell migration and si-TGF-b1 can reserve decreased TPC-1 and SW579 cell migration caused by silencing ANRIL (Figure 5).

**Figure 5:** The migration ability of TPC-1 and SW579 cells in each group by transwell assay after transfection (×200) (**A**) blank group; (**B**) negative control (NC) group; (**C**) si-ANRIL group; (**D**) si-TGF-β1 group; (**E**) si-ANRIL + si-TGF-β1 group; (**F**) Transwell migration histogram of TPC-1 cells in each group after transfection; *, compared with blank group and NC, *P* < 0.05; #,compared with si-ANRIL group, *P* < 0.05.

### Silencing ANRIL expression inhibits TPC-1 and SW579 cell invasion

The numbers of cells invaded through membranes in the blank group and the NC group were 55.6 ± 7.8 and 46.31 ± 5.12, the NC group were 54.8 ± 6.5 and 43.62 ± 5.28, and si-ANRIL group were 30.5 ± 5.7 and 19.43 ± 3.52, respectively. The number of cells invaded through membranes in the si-ANRIL group was lower relative to the blank group and the NC group (both *P* < 0.05), while the number of cells invaded through membranes between the blank group and the NC group was not significantly different (*P* > 0.05). Silencing ANRIL can inhibit the invasion of TPC-1 and SW579 cells; the number of cells invaded through membranes in the si-TGF-β1 group were 100.3 ± 9.2 and 86.34 ± 6.24, and the si-ANRIL + si-TGF-β1 group were 89.2 ± 8.9 and 70.59 ± 5.36, respectively, both of which were significantly higher relative to the blank group and the NC group (all *P* < 0.05). These findings suggested that silencing TGF-β1 can promote the invasion ability of TPC-1 and SW579 cells, and TGF-β1 siRNA can reverse decreased invasion ability of TPC-1 and SW579 cells induced by si-ANRIL siRNA (Figure 6).

**Figure 6:** The invasion ability of TPC-1 and SW579 cells in each group by transwell assay after transfection (×200) (**A**) blank group; (**B**) negative control (NC) group; (**C**) si-ANRIL group; (**D**) si-TGF-β1 group; (**E**) si-ANRIL + si-TGF-β1 group; (**F**) Transwell invasion histogram of TPC-1 cells in each group after transfection; *, compared with blank group and NC, *P* < 0.05; #,compared with si-ANRIL group, *P* < 0.05.

### Effects of silencing ANRIL on p15^INK4b^, p14^ARF^ and p16^INK4a^ expressions in TPC-1

The qRT-PCR was applied to detect the regulatory role of ANRIL in the INK4b/ARF/INK4a encoded tumor suppressor genes p15^INK4b^, p14^ARF^ and p16^INK4a^ in TPC-1 and SW579 cells. As presented in Figure 7, the si-ANRIL group showed higher expression of p15INK4b mRNA than the blank group and the NC group (both *P* < 0.05), and there was no statistical difference in p15INK4b mRNA expression between the blank group and the NC group (*P* > 0.05); the si-TGF-β1 group and the si-ANRIL + si-TGF-β1 group had significantly lower p15INK4b mRNA expressions than the blank group and the NC group (all *P* < 0.05); p14ARF and p16INK4a mRNA expressions in the si-ANRIL group were significantly higher than those in the blank group and the NC group (all *P* < 0.05), but the si-TGF-β1 group or the si-ANRIL + si-TGF-β1 group showed no significant difference in p14^ARF^ or p16^INK4a^ mRNA expressions compared with the blank group and the NC group (all *P* > 0.05). Thus the silencing of TGF-β1 expression blocked the inhibitory effect of ANRIL silencing on p15^INK4b^.

**Figure 7:** The mRNA expressions of tumor suppressor genes p15^INK4b^ (A) p14^ARF^ (B) and p16^INK4a^ (C) detected by qRT-PCR; *, compared with the blank group and NC group, *P* < 0.05; #, compared with si-ANRIL group, *P* < 0.05 qRT-PCR, quantitative real-time polymerase chain reaction.

### ANRIL acts through TGF-β/Smad signaling pathway

In order to verify whether the ANRIL inhibits the expression of tumor suppressor gene p15^INK4b^ through TGF-β/Smad signaling pathway, the expressions of TGF-β1 and downstream key protein p-Smad2/3 in the TGF-β/Smad signaling pathway were detected with western blot. Western blot results showed that 24 h after ANRIL siRNA transfection, TGF-β1 and p-Smad2/3 expressions in TPC-1 and SW579 cells were up-regulated compared with the blank group and the NC group (both *P* < 0.05), TGF-β1 and p-Smad2/3 expressions in the si-TGF-β1 group and the si-ANRIL + si-TGF-β1 group were significantly lower than those in the blank group and the NC group (all *P* < 0.05); no differences in TGF-β1 and p-Smad2/3 expressions were found between the blank group and the NC group (all *P* > 0.05), as shown in Figure 8.

**Figure 8:** ANRIL acts through TGFβ/Smad signaling pathway: the expressions of TGF-β1 (**A**) effects of ANRIL siRNA transfection on TGF-β1 protein level in TPC-1 and SW579 cells detected by Western blot; (**B**) p-Smad2/3 protein expression in the TPC-1 and SW579 cells in each group detected by Western blot; *, compared with blank group and NC, *P* < 0.05; #, compared with si-ANRIL group, *P* < 0.05.

### Visceral metastasis

Transwell invasion and migration experiments have shown that ANRIL has a certain influence on the invasion and migration of TPC-1 cells. The visceral metastasis experiment results showed that mice injected with ANRIL siRNA transfected TPC-1 cells had significantly decreased lung metastatic nodules compared with the NC group and the blank group. The number of lung metastatic nodules in the si-ANRIL group was lower relative to the NC group and the blank group (both *P* < 0.01). Therefore, ANRIL silencing can inhibit visceral metastasis of TPC-1 cells. Mice injected with TGF-β1 siRNA transfected TPC-1 cells had significantly increased lung metastatic nodules compared with the NC group and the blank group (both *P* < 0.05). The number of lung metastatic nodules in the si-ANRIL + si-TGF-β1 group was markedly higher in comparison to the si-ANRIL group (*P* < 0.05) (Figure 9A–9E). The evidence indicated that the silence of TGF-β1 can promote visceral metastasis ability of TPC-1 cells and TGF-β1 siRNA can reverse si-ANRIL siRNA caused declined visceral metastasis ability of TPC-1 cell. The average value of visible nodules was shown in Figure 9F.

**Figure 9:** HE staining (A–E) and statistical analysis (F) results of lung metastatic nodules in the nude mice after tail vein injection of TPC-1 cells (× 200) (**A**), blank group; (**B**), negative control (NC) group; (**C**) si-ANRIL group; (**D**) si-TGF-β1 group; (**E**) si-ANRIL + si-TGF-β1 group; (**F**) statistical analysis of lung metastatic nodules in the nude mice; *, compared with blank group and NC, *P* < 0.05; #,compared with si-ANRIL group, *P* < 0.05; LM, lung metastasis.

## DISCUSSION

In the present study, the TC tissues are presented with significantly higher relative expression of ANRIL mRNA than the adjacent normal tissues. Significant differences in the relative expression of ANRIL mRNA were found for TNM stages and LNM, suggesting that ANRIL may play a carcinogenesis role in TC. It has been previously described that aberrant lncRNA expression may contribute to tumorigenesis, and a genome-wide analysis of lncRNA expression profile in TC provides a reference for further assessing TC related lncRNAs [23, 24]. Moreover, the roles of lncRNAs in TC development have been highlighted in recent studies: PTCSC3 was involved in TC development by modulating S100A4 gene expression, NONHSAT037832 might serve as a potential biomarker of TC, and FAL1 might play certain roles in cell-cycle progression and aggressive tumor behavior in TC [25–28]. With respect to ANRIL, significantly increased expressions of ANRIL have been found in cancer tissues including serous ovarian cancer (SOC), hepatocellular carcinoma (HCC), bladder cancer, ESCC and non-small-cell lung cancer, further, clinicopathologic significances of the ANRIL expressions have been found regarding clinical stage, histological grade, LNM, tumor size [18, 19, 29–31]. However, the expression of ANRIL and the involvement of ANRIL in the development of TC failed to be well studied. This research found that the adjacent normal tissues have significantly higher positive rate of TGF-β1 expression than the TC tissues, and TGF-β1 expression may be associated with clinical stage and LNM of TC. Higher expression levels of TGF-β1 and the close relationship of TGF-β1 and LNM in TC have been reported in increasing evidence, indicating that immunohistochemical and RT-PCR evaluation of TGF-β1 expression may be useful to predict the risk of LNM in TC [21, 32, 33]. Furthermore, our spearman correlation analysis showed that the ANRIL expression was positively correlated with the expression of TGF-β1 protein expression.

The qRT-PCR results demonstrated that lncRNA ANRIL is highly expressed in the TC cell line compared with the normal thyroid cell lines, and further experiments were carried using TPC-1 cell line as a model cell to study the function of ANRIL in TC. The siRNA-mediated ANRIL silencing significantly inhibited the growth, migration and invasion, as well as visceral metastasis of TPC-1 cells; while siRNA-mediated TGF-β1 silencing can reverse the ANRIL siRNA induced inhibition of growth, migration and invasion, as well as visceral metastasis of TPC-1 cells. LncRNAs played functional roles in controlling gene transcription through targeted recruitment of epigenetic silencing complexes to genomic homology-containing loci [13]. The siRNA-mediated ANRIL silencing in SOC cells impaired cell migration and invasion, and lncRNA ANRIL may have played a significant role in SOC invasion/metastasis [29]. Several studies reported that the silencing of ANRIL expression could repress proliferation and invasion and induce apoptosis in different cancer cells [18, 30, 31]. Depletion of ANRIL by transfected with ANRIL siRNAs caused cell-cycle arrest at the G2/M phase, which led to an inhibition of proliferation of cancer cells via regulating p15 and other genes related to G2/M phase control [34]. ANRIL was transcribed in the opposite direction from INK4b-ARF-INK4a gene cluster encoding three tumor suppressors: p15(INK4b), p14(ARF), and p16(INK4a), and it has been suggested that ANRIL repressed the expression of p15(INK4b), p14(ARF), and p16(INK4a) [19]. In our study, siRNA-mediated ANRIL silencing resulted in up-regulated p15^INK4b^, p14^ARF^ and p16^INK4a^ mRNA expressions, while siRNA-mediated TGF-β1 silencing led to down-regulated p15^INK4b^ mRNA expression, suggesting that silencing of TGF-β1 expression can block the inhibitory effect of ANRIL silencing on p15^INK4b^. Accumulating evidence suggested important role of TGF-β1/Smad signaling pathway in TC development, such as cell differentiation, tumor invasion, etc. [21, 35–37]. In order to investigate the possible mechanisms underlying lncRNA expression changes and TC, we conducted further experiments to verify whether the ANRIL decreases the expression of tumor suppressor gene p15INK4b through TGF-β/Smad signaling pathway. The results indicated that ANRIL may decrease the expression of p15^INK4b^ through inhibiting TGF-β/Smad signaling pathway, promoting the invasion and metastasis of TC cells. As previously described, Chen D *et, al*. suggested that ANRIL inhibited p15(INK4b) possibly through the TGF-β1 signaling pathway, and played functional roles in human ESCC [19]. ANRIL is transcribed in the opposite direction from the INK4b-ARF-INK4a gene cluster that encodes three tumor suppressors: p15^INK4b^, p14^ARF^, and p16^INK4a^ [38]. ANRIL has been reported to be involved in cancer cell proliferation by silencing p15^INK4^ expression. Therefore, it is plausible to propose that the mechanisms involved by ANRIL in the down-regulation of TGF-β signaling and cell growth and migration may be explained by that ANRIL can promote the invasion and metastasis of TC cells by reducing p15^INK4B^ expression through inhibiting TGFTGF-β/Smad signaling pathway.

Furthermore, in order to further verify our results *in vitro*, we constructed xenograft tumor in nude mice to compare lung metastasis. The results showed that mice injected with ANRIL siRNA transfected TPC-1 cells had significantly decreased lung metastatic nodules compared with the NC group and the blank group, and the number of lung metastatic nodules in the si-ANRIL group was lower relative to the NC group and the blank group, suggesting that ANRIL silencing can inhibit visceral metastasis of TPC-1 cells. In addition, mice injected with TGF-β1 siRNA transfected TPC-1 cells had significantly increased lung metastatic nodules compared with the NC group and the blank group, and the number of lung metastatic nodules in the si-ANRIL + si-TGF-β1 group was markedly higher in comparison to the si-ANRIL group, indicating that the silence of TGF-β1 can promote visceral metastasis ability of TPC-1 cells and TGF-β1 siRNA can reverse si-ANRIL siRNA caused declined visceral metastasis ability of TPC-1 cells. Therefore, visceral metastasis findings in the rat experiment further improve the credibility of our above results and provide a clinical significance for ANRIL and TGF-β/Smad signaling pathway in TC.

In conclusion, and the silencing ANRIL, as a key lncRNA, inhibits the invasion and metastasis of TPC-1 cells. Moreover, ANRIL may inhibit the expression of TGF-β/Smad signaling pathway to reduce p15^INK4B^ expression and promote invasion and metastasis of TC cells, which provides a novel insight on the functional role of lncRNA ANRIL-driven tumorigenesis. However, due to our limitation in time and funds, further experiments which may contribute to the understanding of the molecular mechanisms that may be involved in the ANRIL dependent regulation of TGF-β1 signaling pathway and the biological features described were not performed, and we only collected samples from cancer tissues and adjacent tissues rather than normal tissues. In the future, these experiments with larger sample size from cancer tissues, adjacent tissues as well as normal tissues will be further conducted when conditions permit to improve our preliminary work and clarify the molecular mechanisms in depth.

## MATERIALS AND METHODS

### Sample collection

From March 2013 to March 2015, 105 TC patients who received surgical treatment in the Department of Thyroid and Breast Surgery in Research Institute of Surgery, Daping Hospital, and Third Military Medical University were recruited. TC was confirmed by postoperative pathological diagnosis. The 105 TC patients include 38 males and 67 females with a mean age of 52.0 ± 11.2 years (age range, 29–82 years). The 105 TC patients were mainly presented with neck mass (solitary nodule in 78 cases, multiple nodules in 13 cases) and hoarse voice (14 cases), and clinically palpable hard masses with unclear boundaries and no obvious tenderness. All patients underwent surgical treatment, and the tumor tissues and the adjacent normal tissues (thyroid tissues > 5 cm from the margin of the tumor) were resected during surgery as paired samples. Tissue samples were immediately put into liquid nitrogen for rapid freezing, and transferred to a −80 DEG ultra-low temperature refrigerator for further usage. The tissue samples were divided into 2 parts, one was used for the detection of lncRNA ANRIL, and the other was fixed with 10% formaldehyde and embedded in paraffin for the detection of protein expression of TGF-β1 by immunohistochemistry (ICH).

Patients were included if they were confirmed by pathology, and were not treated with iodine 131, thyroid stimulating hormone suppression or radiotherapy before admission. Patients were excluded if they: received iodine 131 or thyroid stimulating hormone inhibition therapy before surgery; have incomplete clinical or pathological data, such as the lack of pathological diagnosis report or lack of lymph node metastasis (LNM) related inspection report; combined with other malignant tumor; had malignant tumor with distant metastasis to the thyroid gland; suffered from serious systemic infections or other severe systemic diseases. All the patients and signed informed consent. The experiment protocol was approved by the ethics committee of clinical laboratory.

### Cell culture

Human papillary thyroid cancer cell line K1 and TPC-1, human thyroid squamous cell carcinoma cell line SW579 and human thyroid cell line Nthy-ori 3–1 purchased from American Type Culture Collection (ATCC) were cultured in DMEM medium with 10% fetal bovine serum (FBS), and incubated in incubator with 5% CO_2_ at 37°C. Cells shown monolayer growth and cell passage was carried out when the cell attachment rate reach 90%. Cells were conventionally passaged, and the primary medium was moved. Cells were washed two times with PBS and digested in 0.25% trypsin, and the 0.25% trypsin was removed after increased intercellular space was observed. Finally, cells were made into single cell suspension using RPMI-1640 medium containing calf serum with a volume fraction of 10%.

### Cell grouping and transfection

Cells were randomly divided into si-ANRIL group (transfected with si-ANRIL), si-TGFβ1 group (transfected with si-TGF-β1), si-ANRIL + si-TGF-β1 group (co-transfected with si-ANRIL + si-TGF-β1), negative control (NC, transfected with NC sequence) group and blank group (transfected with no sequence). TPC-1 and SW579 cells were inoculated into 6-well culture plate for 1 day before transfection (5 × 10^5^ per well) to ensure the confluence reached 80%–90% within 24 h. In accordance with Lipofectaminetm 2000 (Invitrogen) operating instructions, the plasmid and Lipofectaminetm 2000 were added to 250 μL of Opti-MEM, respectively, standing at room temperature for 5 min, the plasmid and Lipofectaminetm 2000 were mixed evenly, after standing for 20 minutes, 500 μL of plasmid /Lipofectamine^TM^2000 mixture was dropped into the 6-well culture plate, and incubated for 48–72 h for follow-up experiments. All transfection sequences were purchased from Invitrogen.

### Quantitative real-time polymerase chain reaction (qRT-PCR)

Total RNA expression of cell liquid to be tested was extracted according to kit specification (Promega), and 5 μl of RNA samples was diluted (× 20) with RNase free ultrapure water, absorption values at 260 nm and 280 nm were read with ultraviolet spectrophotometer to determine the concentration and purity of RNA, with the OD260/OD280 ratio of 1.7–2.1 indicating high purity. RNA was subjected to reverse transcription for cDNA preparation. ABI7500 quantitative PCR instrument was applied to qRT-PCR with the following reaction conditions: pre-denaturation at 95°C for 10 min, degeneration at 95°C for 10 s, anneal at 60°C for 20 s, extension at 72°C for 34 s, 40 cycles. Primer sequences were synthesized by Sangon Biotech (Shanghai) Co., Ltd. and summarized in Table 2. PCR results were analyzed to obtain Ct values of amplified products, and data was analyzed by adopting 2^-ΔΔCt^ method [39], with 2^-ΔΔCt^ demonstrating the relative expression ratios of the target gene of the case group to the control group (ΔΔCt = ΔCt _case group_ - ΔCt _control group_, ΔCt = Ct _target gene_ - Ct _internal reference gene_), Ct (threshold cycle) is the number of amplification cycles when the real time fluorescence intensity of the reaction reaches the threshold values. The amplification was performed during a period of logarithmic growth. The experiment was triplicate.

**Table 2:** Primer sequence

Gene	Primer sequence
lncRNA ANRIL	F: 5′-TGCTCTATCCGCCAATCAGG-3′
	R: 5′-GGGCCTCAGTGGCACATACC-3′
p14ARF	F: 5′-GGCCCTCGTGCTGATGCTAC-3′
	R: 5′-TGGAGCAGCAGCAGCTCCGC-3′
p16 INK4a	F: 5′-CTGCCCAACGCACCGAATAG-3′
	R: 5′-CAGCACCACCAGCGTGTCC-3′
p15INK4b	F: 5′-CGGGGACTAGTGGAGAAGGT-3′
	R: 5′-CGAAACGGTTGACTCCGTTG-3′
GADPH	F: 5′-GTCAACGGATTTGGTCTGTATT-3′
	R: 5′-AGTCTTCTGGGTGGCAGTGAT-3′

### Immunohistochemistry

The expression of TGF-β1 protein was detected by two-step immunohistochemical staining with PV9000 and 3,3′-Diaminobenzidine tetrahydrochloride (DAB). The paraffin-embedded specimens were continuously cut into slices with a thickness of 4 μm. The tissue slices were performed with conventional xylene dewaxing, dehydrated in graded alcohol, followed by microwave thermal antigen repair, block endogenous peroxidase with 3% hydrogen peroxide, and incubated with the primary antibody (rabbit anti human TGF-β1 monoclonal antibody, 1:100) overnight at 4°C. The tissue slices were incubated with polymerase auxiliary agent for 20 min at room temperature, and additionally incubated with the horseradish peroxidase labeled secondary antibody (Beijing Biosynthesis Biotechnology Co. Ltd.) for 30 min at room temperature. Color development was performed with DAB followed by hematoxylin redyeing and mounting. The negative control was prepared by replacing the primary antibody with PBS, and normal mucosa tissues were used as the positive control. The expression of TGF-β1 was mainly observed in kytoplasm and cytomembrane, and presented with yellow or brownish granules. Five high-power fields (400×, 100 cells per field) in each tissue slice were randomly selected, and positive cells/all tumor cells > 10% was considered as positive (+) and positive cells ≤ 10% as negative (−). The results of immunohistochemistry were evaluated independently by two experienced observers in a double blind method.

### Methyl thiazolyl tetrazolium (MTT) colorimetry

Cells were washed with PBS twice when grown to confluence (80% confluent). Cells were inoculated in a 96-well plate (200 μl per well, 6 repeated wells) in a density of 3 × 10^3^ ~ 6 × 10^3^. Cells were incubated at 37°C, 5% CO_2_ for 24–72 h, and 20 μl of MTT solution (5 mg/ml, Sigma) were added into each well. After 4 h incubation at 37°C and 5% CO_2_, the incubation was terminated, and the culture medium was discarded. DMSO (150 μl) (Sigma) was added to each well, and gently shaken for 10 min to promote crystallization dissolution. Absorbance values (OD) were determined with an enzyme-linked immunosorbent detector at 12 h, 24 h and 48 h, respectively. MTT curve was draw with interval time as the X-axis and the OD value as the Y-axis. The experiment was triplicated.

### Cell counting

Well-grown transfected cells were inoculated in a 24-well plate in a density of 1 × 10^4^; after cultured for 24 hours and digested with 0.25% trypsin, cell suspension was made; 10 ul cell suspension was placed in the cell counting plate for counting; each hole was repeated three times for the average value to reflect the cell proliferation. Original cell number/ul = (four large cell number /4) ×10^4^.

### Transwell for the detection of cell migration and invasion

TPC-1 and SW579 cells in the logarithmic growth phase were cultured in serum free medium for 24 h and digested. The cell density was adjusted to 3 × 10^4^/ml with serum free medium. Cell suspension with adjusted cell density (100 μl) was added into the upper chamber, culture medium (500 μl) containing 10% FBS was added into the lower chamber and Transwell chambers were covered and incubated. The upper chamber was removed to 24-well Transwell plates, marked, covered and then incubated. The culture medium in the upper chamber was removed and 4% formaldehyde (600 μL) was added into the 24-well Transwell plates. The upper chamber was then moved to wells containing 4% formaldehyde, and anhydrous methanol (150 μL) was added. The upper chamber was marked, the anhydrous methanol in the upper chamber was removed after 15 min standing, and the upper chamber was inverted on covers of the 24 -well Transwell plates. The lower surface of the upper chamber was air-dried naturally in a ventilated kitchen. Giemsa reagent 1 was added into the upper chamber, standing for 1 min, then Giemsa reagent 2 was added into the upper chamber, standing for 5 min. After this, the upper chamber was washed with PBS (30 min/3 times), results were observed and photographed under the inverted microscope, and were further observed and photographed with a microscope image acquisition system. Five field counts were randomly selected. In invasion test, the number of cells in each group passing through the Matrigel was used as an index for evaluating the ability of invasion, and the migration test without adding the Matrigel shared the same steps with the invasion test.

### Western blot

The total protein was extracted according to the instructions of the total protein extraction kit (Beijing solarbio science and technology co., Ltd.). Total protein content was determined by BCA method. The total protein was run on 12% SDS-PAGE (sample size, 50 μg) and electro-transferred to nitrate cellulose (NC) membranes. The membranes were blocked with 5% skim milk, incubated with commercially purchased antibodies to TGF-b (Cell Signaling Technology; Boston, Massachusetts, USA), phosphorylated Smad2/3 (p-Smad2/3; Ser 423/425; Santa Cruz Biotechnology;Santa Cruz, CA, USA) and β-actin (CWBIO; Beijing, China) overnight at 4°C. After this, they were washed with TBST (3 times, 10 min/time), incubated with secondary antibody at room temperature for 1 h, and further washed with TBST (3 times, 10 min/time). Finally, the processes of chemiluminescence, X ray film processing, developing and fixing and data analysis were carried out.

### Visceral metastasis from the tail vein of nude mice

Female nude mice (*n* = 50) (purchased from the Animal Center of Chinese Academy of Medical Sciences, Beijing) were housed in constant humidity (45%–50%) and constant temperature (25–27°C). Sterilized water and feed were provided *ad libitum*. The nude mice were divided into five groups, with 10 rats in each group: si-ANRIL group (injected with ANRIL siRNA transfected TPC-1 and SW579 cells), si-TGF-β1 group (injected with TGF-β1 siRNA transfected TPC-1 and SW579 cells), si-ANRIL + si-TGF-β1 group (injected with ANRIL siRNA and TGF-β1 siRNA transfected TPC-1 and SW579 cells), NC group (injected with NC transfected TPC-1 and SW579 cells) and blank group (injected with untransfected TPC-1 and SW579 cells). The experimental program was approved by the ethics committee of the animal experimental center of Daping Hospital, Third Military Medical University and combined with the ethical principles of animal experiments established in 1996 by The National Institutes of Health (NIH).

When cell density grew to about 80%–90% with good state, the cells were digested and resuspended, and the number of cells was counted. The concentration of cell suspension was adjusted to 1 × 10^7^/ml; the tail vein of each mouse was injected with 0.2 ml of cell suspension containing about 2 × l0^6^ cells. Each cell line was inoculated into 10 nude mice, and mice were observed 3–4 times per week. After feeding for 6–7 weeks, mice were killed, the lungs were removed, rinsed with physiological saline to remove the blood, and put into formaldehyde [40]. Hematoxylin and eosin (H&E) staining was carried out for the analysis of lung metastasis.

### H&E staining

Lung biopsies of nude mice were performed with dewaxing in xylene for 5–10 minutes, put into xylene and pure alcohol (1:1) mixture for 5 minutes, followed by 100%, 95%, 85%, 70% graded alcohol for 2–5 minutes, distilled water and dye. Lung biopsies were subjected to hematoxylin stain for 5–15 minutes, and unnecessary dye was washed; 1% hydrochloric acid alcohol (prepared by 70% alcohol) was used for color separation, and microscopic control was performed until the nucleus and nuclear chromatin were clear (about 10 seconds), the Lithium carbonate saturated liquid was used for alkalizing or bluing the cells in a short period of time, namely until the nucleus turned blue. Lung biopsies were washed the distilled water for a short while, and stained with 0.3% eosin for 1–5 minutes. When coloring became problematic, 1–2 drops of acetic acid were added into the dye per 100 ml to make it easy to color and not easy to discolor. Lung biopsies were treated with 70%, 85%, 95% and 100% alcohol dehydration (3 min for each grade), and since eosin easily discolors in alcohol below 95% in alcohol, time was appropriately shorten. Lung biopsies were transparent by xylene (twice) for 10 min, and sealed with neutral gum. The number of lung nodules was observed under optical microscope.

### Statistical analyses

SPSS 19.0 software (SPSS Inc., Chicago, IL, USA) was used for statistical analysis. Data was presented as means ± standard deviation (SD). Multi group comparisons were performed with one-way ANOVA after homogeneity test of variance, and LSD-*t* test for pairwise comparison. Spearman correlation analysis was applied to show the correlation between the expression level of lncRNA ANRIL and TGF-β1. A *P* value of < 0.05 indicated statistical significance.
